The article "Effect of Arthroscopic Acromioplasty Combined with Rotator Cuff Repair in the Treatment of Aged Patients with Full-Thickness Rotator Cuff Tear and Rotator Cuff Injury" was retracted in 2024. Reasons: signs of a paper mill; suspected computer-generated content; unreliable results or conclusions; concerns about the data.

# Effect of Arthroscopic Acromioplasty Combined with Rotator Cuff Repair in the Treatment of Aged Patients with Full-Thickness Rotator Cuff Tear and Rotator Cuff Injury

**DOI:** 10.1155/2022/4475087

**Published:** 2022-08-03

**Authors:** Shihui He, Hao Xu, Shuhua Liu

**Affiliations:** Department of Orthopaedics, Zhoushan Hospital, Zhoushan, Zhejiang Province 316000, China

## Abstract

Full-thickness rotator cuff tear and rotator cuff injury are frequently occurring diseases and widely exist in the social population. Surgical repair is the most effective treatment for rotator cuff tears and injuries. With the continuous development of arthroscopy, more and more surgeons choose arthroscopic acromioplasty plus rotator cuff repair for the treatment of rotator cuff injury. However, previously published systematic reviews or meta-analyses still cast doubt on the efficacy of such concomitant procedures for postoperative patient function and pain recovery. In this study, we analyzed the effects of parameters such as shoulder function and acromion morphology on aged patients with full-thickness rotator cuff tear combined with rotator cuff injury treated with arthroscopic acromion plasty and rotator cuff repair. The results showed that arthroscopic acromion plasty and rotator cuff repair helped to promote the joint function recovery of the aged patients with full-thickness rotator cuff tear combined with rotator cuff injury and alleviate the pain of the patients. Compared with simple rotator cuff repair, this technique can increase the postoperative AT and reduce the ACEA and to some extent reduce the risk of postoperative rotator cuff reinjury, which is worthy of promotion.

## 1. Introduction

Full-layer rotator cuff tear and rotator cuff injury are common shoulder joint diseases in clinics, mainly causing shoulder pain and dysfunction. Rotator cuff injury is a common disease in the elderly and one of the main causes of shoulder pain and dysfunction in the elderly. If not treated in time, it will seriously affect the quality of life of patients [1]. There are mainly conservative treatments and surgical treatments for full-thickness rotator cuff tear and rotator cuff injury [2]. Among them, surgical treatments include open rotator cuff repair, arthroscopically assisted small incision rotator cuff repair, and full arthroscopic rotator cuff plasty. Since Codman first proposed rotator cuff injury in 1911, open rotator cuff repair has become the “gold standard” for the treatment of rotator cuff injury [3]. However, with the development and promotion of arthroscopy, arthroscopic repair of the shoulder has become the main treatment for rotator cuff injury, owning to the advantages of small operation trauma, low postoperative adhesion risk, low infection probability, and easy early rehabilitation after operation [4]. In addition, because most patients with rotator cuff injury have subacromial impingement, that is, the greater tubercle of the humerus will collide with the lower surface of the acromion in the process of shoulder abduction of 60–120 [5]. So, acromioplasty is also particularly important in the treatment of rotator cuff injury. However, some studies have suggested that the combined use of acromioplasty and arthroscopic repair for patients with rotator cuff injury is of little significance due to the reproducible morphological structure of the acromion [6]. The value of the combined use of these two procedures remains controversial. On this basis, this study explored the effects of arthroscopic acromioplasty plus rotator cuff repair on the shoulder function and acromion morphology of aged patients with full-thickness rotator cuff tear and rotator cuff injury, aiming to analyze the clinical effect of this treatment. The results are now reported as follows.

## 2. Materials and Methods

### 2.1. General Information

All patients with shoulder pain who were admitted to our hospital from January 2019 to June 2020 were selected. Among the patients initially diagnosed with rotator cuff injury by ultrasound examination, 84 patients met the inclusion and exclusion criteria. According to the difference in treatment methods, the patients were divided into a study group and a control group, with 42 cases in each group. This study has been approved by the Hospital Medical Ethics Committee.

### 2.2. Inclusion Criteria

(1) Compliant with the diagnosis of rotator cuff tear combined with rotator cuff injury, and age >60 years old [7]. (2) Patients with indications for rotator cuff repair. (3) No previous operation history of shoulder. (4) No recent infectious disease. (5) The skin is not damaged. (6) Voluntary participation in the study and timely follow-up.

### 2.3. Exclusion Criteria

(1) Patients with shoulder pain and abnormal anatomical structure caused by infection, deformity, and other reasons. (2) Combined with periarticular fractures.(3) Patients who refuse to be interrupted during surgery or treatment and cannot be followed up on time. (4) Coagulation dysfunction. (5) Passive movement of the shoulder joint was performed to confirm the surgical effect.

### 2.4. Method

Patients in the study group underwent arthroscopic acromioplasty plus rotator cuff repair. The surgical procedures were as follows: after the patient's endotracheal general anesthesia was successful, the healthy lateral decubitus position was taken. The body is reclined 20°, the shoulder joint abduction is 45–60°, and the anterior flexion is 15–20°. Abduction of the affected shoulder joint is 45–60°. Limb sleeve set good, with a bandage and film. Anterior superior flexion of the healthy limb was performed to maintain the mild abduction, anterior flexion, and traction state of the affected upper limb. The affected limb was suspended by the shoulder arthroscopic traction device. The systolic blood pressure was controlled to 90–100 mmHg during the operation. After the acromion, coracoid process, and scapular ridge were marked, the operation fields were disinfected and draped. Normal saline was first injected into the shoulder joint to expand the joint capsule. Then, a posterior approach to the shoulder was selected for puncture, followed by continuous irrigation with epinephrine normal saline (3,000 mL of normal saline plus 1 mL of epinephrine). After a thorough examination of the glenohumeral joint, the arthroscopic sheath and blunt round trocar were repositioned in the subacromial space. A plane knife was inserted through the anteromedial approach to the acromion to clear the glide sac of the acromion and fully expose the lower surface of the acromion and the coracoacromial ligament. Carefully explore the shape of the anterior outer edge of the acromion. Anterior and posterolateral approaches were established. The rotator cuff tear was observed, and the injury margin of the supraspinatus tendon was explored. According to the size of the tear, the quality of humerus bone, and the condition of the suture port, double rows of anchors were used to strengthen the suture. Stop bleeding, and move the shoulder joint. After the examination and repair were satisfactory, the wound was fully sutured. During the operation, a grinding drill was used to grind the anterior 1/3 bone cortex of shoulder peak to a depth of about 4 mm and a width of about 10 mm. After that, passive movement of the shoulder joint was performed to confirm the surgical effect.

Patients in the control group were treated with simple arthroscopic rotator cuff repair, and the operation procedures were the same as those in the study group.

All the patients received routine anti-infection treatment 24 h after operation, and the drainage tube was removed within 48 h after operation. Meanwhile, procedural rehabilitation was performed by the same rehabilitation physician according to the same principles of rehabilitation treatment.

### 2.5. Observation Indicators

1. Shoulder joint function: all patients received shoulder joint function scoring examination before operation and 6 months after operation. Constant–Murley shoulder joint scoring system and UCLA shoulder joint scoring system were used as scoring tools. The Constant–Murley shoulder joint scoring system was divided into four aspects including pain, arm posture, range of motion, and abduction muscle strength, with scores ranging from 0 to 100 points [8]. The UCLA shoulder joint scoring system was divided into five aspects, i.e., pain, function, active upper limb anteflexion, upper limb anteflexion muscle strength, and patient satisfaction. The full score was 35 points, and a score less than 27 points indicated that the recovery was not ideal [9].
2. Pain conditions: two groups were assessed with visual analogue scales (VAS) before operation, 2 weeks after operation, 2 months after operation, and 6 months after operation. According to clinical evaluation, “0–2” was classified as “no pain or almost negligible,” “3–5” as “mild pain,” “6–8” as “moderate pain,” and “8” as “severe pain” [10].
3. Active range of motion of affected shoulder: the range of motion of affected shoulder flexion, abduction, neutral external rotation, abduction 90 internal rotation, and abduction 90 external rotation of the two groups were evaluated before operation and six months after operation.
4. Morphological parameters of acromion: standard anteroposterior radiographs of the shoulder were taken before and six months after the operation, and the critical shoulder angle (CSA), acromial tilt angle (AT), lateral acromion angle (LAA), acromion index (AI), and acromiohumeral centre edge angle (ACEA) were recorded. Among them, CSA angle refers to the angle formed by the angle between the upper and lower edges of glenoid fossa and the lower edge of glenoid fossa to the outermost lower edge of acromion. AT was the line connecting the rearmost point and the forwardmost point of the lower margin of acromion and the line connecting the rearmost point of the lower margin of acromion and the lower margin of coracoid process, respectively. LAA was the angle between the line connecting the outermost upper and lower edges of the glenoid and the line connecting the lower surface of the acromion. AI refers to the ratio of the distance between the glenoid plane and the lateral surface of the acromion to the distance between the glenoid plane and the lateral surface of the humeral head. ACEA refers to on the positive X-ray film of shoulder joint, the circle with the largest area covering the whole humeral head was firstly simulated according to the articular surface of humeral head, the line between the midpoint of this circle and the outermost point of acromion, and the angle between this line and the parallel line of glenoid across the circular midpoint.
5. The operation time, bleeding volume, incision length, and length of hospital stay were compared between the two groups.
6. The complications such as vascular and nerve injury, postoperative infection, postoperative joint adhesion, and retear were compared between the two groups.

### 2.6. Statistical Methods

All data were processed with SPSS 22.0 statistical software, and GraphPad prism 8 was used to make statistical graphs. Measurement data are expressed as mean ± standard deviation ($\bar{x}$ ± *s*), independent sample *t*-test is used for comparison between groups, count data is expressed as *n* (%), and chi-square (*χ*^2^) test is performed. The difference is statistically significant when *P* < 0.05.

## 3. Results

### 3.1. Baseline Data

There was no significant difference in general data between the two groups, which was comparable (*P* > 0.05, Table 1).

### 3.2. Comparison of Constant–Murley and UCLA Scores before and after Surgery in Two Groups

There was no significant difference in the Constant–Murley score and UCLA score between the two groups before operation (*P* > 0.05). After surgery, the Constant–Murley scores and UCLA scores in the two groups were higher than those before surgery, and the scores in the study group were higher than those in the control group (*P* < 0.05, Table 2).

### 3.3. Comparison of VAS Scores of Patients between the Two Groups before and at Each Time Point after Surgery

There was no significant VAS score between the two groups before operation (*P* > 0.05). The VAS scores of the patients in the two groups two weeks after the operation, two months after the operation, and six months after the operation were lower than those before the operation, and the VAS scores of the patients in the study group at each time point after the operation were lower than those in the control group (*P* < 0.05, Table 3).

### 3.4. Comparison of Active Range of Motion between the Two Groups before and after Surgery

There was no significant difference in the range of motion of preoperative shoulder flexion, abduction, neutral external rotation, abduction 90 internal rotation, and abduction 90 external rotation between the two groups (*P* > 0.05). After surgery, the range of motion of anterior shoulder flexion, abduction, neutral external rotation, abduction 90 internal rotation, and abduction 90 external rotation in both groups were significantly increased as compared with those before surgery, and the range of motion in the study group was higher than that in the control group (*P* < 0.05, Table 4).

### 3.5. Comparison of Morphological Parameters of Acromion between the Two Groups before and after Surgery

Before surgery, the comparisons of CSA, AT, LAA, AI, and ACEA between the two groups were not statistically significant (*P* > 0.05). After surgery, CSA decreased, AT increased, and ACEA decreased in both groups (*P* < 0.05), but LAA and AI were not different from those before surgery. After surgery, CSA and ACEA levels in the treatment group were smaller than those in the control group, and AT level was larger than that in the control group (*P* < 0.05, Table 5).

### 3.6. Comparison of Surgical Indexes between the Two Groups

The length of hospital stay in the study group was shorter than that in the control group (*P* < 0.05). However, the operation time, blood loss, and incision length between the two groups were not statistically significant (*P* > 0.05, Table 6).

### 3.7. Comparison of Postoperative Complications between the Two Groups

There was 1 postoperative infection in the study group and 1 postoperative joint adhesion in the control group. There was no statistical significance in the incidence of complications between the two groups (*P* < 0.05).

## 4. Discussion

At present, it is considered that the causes and pathogenesis of full-thickness rotator cuff tear and rotator cuff injury include advanced age, trauma, rotator cuff blood supply insufficiency, chronic impingement injury of the rotator cuff, and rotator cuff degeneration [11]. Nowadays, arthroscopic rotator cuff repair is widely used; however, in the research on the treatment of rotator cuff injury, with the proposal of the theory of subacromial impingement, researchers have paid attention to the effect of acromion morphology on the degree of rotator cuff injury [12, 13]. Acrominoplasty has become an auxiliary project of arthroscopic rotator cuff repair [14].

This study showed that, after surgery, the Constant–Murley and UCLA scores of patients in the study group were higher than those of the control group, and the VAS score was lower than that of the control group. Moreover, the joint range of motion of patients in the study group was also superior to that of the control group (*P* < 0.05). This indicates that arthroscopic acromioplasty plus rotator cuff repair is conducive to promoting the joint function recovery of elderly patients with full-thickness rotator cuff tear combined with rotator cuff injury and reducing the pain in the patients. Acromioplasty is defined as a surgery in which the osteophytes on the anterior and inferior border of the acromion are excised so that the type II and III acromions can be converted into type I acromion [15]. We believe the clinical advantages of acromioplasty while arthroscopic rotator cuff repair lies in the following aspects: ① performing acromioplasty before repair of a damaged rotator cuff can change the morphology of the acromion and reduce the rate of postrepair injury of rotator cuff injury due to the acromion impingement sign [16]. ② Acrominoplasty can clean the glide sac of acromion that can cause pain, alleviate the pain, and increase the subacromial space, providing convenience for arthroscopic operation and improving the surgical effect [17]. ③ Acromioplasty has little effect on the deltoid muscle, and it can increase the expression of bone marrow stem cells and related mediators, helping the patient recover faster. ④The injury to the deltoid muscle is small, so that the probability of shoulder joint activity limitation and retearing caused by the deltoid muscle function injury after the operation is reduced [18]. This study showed that the patients in the study group had no postoperative complications such as vascular and nerve injury, postoperative joint adhesion, and retear, confirming the safety of arthroscopic acromioplasty plus rotator cuff repair.

The purpose of rotator cuff repair is to anatomize and reconstruct the stop point of the rotator cuff, so as to minimize the pain of patients and restore their joint function. Previous studies have reported that the absence of simultaneous acromioplasty during rotator cuff repair increases the risk of rotator cuff reoperation [19]. Therefore, in this study, the morphological parameters of the acromion in patients undergoing arthroscopic rotator cuff repair together with acromioplasty were measured before and after the operation, in order to find out the effect of this surgical scheme on the morphological parameters of the acromion in elderly patients with full-thickness rotator cuff tear combined with rotator cuff injury and further explore the effect of this operation on the risk of rotator cuff reinjury. Previous studies think that CSA >35 would significantly increase the risk of rotator cuff injury [20]. In this study, CSA in both groups was above 35 before the operation, but it was <35 after treatment. Besides, CSA in the study group was smaller than that in the control group after the operation. This indicates that it is obvious that acromioplasty during the operation can change the angle of CSA and reduce the occurrence of rotator cuff reinjury [21]. The decrease in Ming AT is related to the increase in rotator cuff injury. The increase of ACEA suggested that the coverage area of the humeral head covered by acromion was increased [22]. In case of acromion impact, the risk of rotator cuff injury was increased. The results showed that the AT of patients in the study group after surgery was larger than that of the control group, and the ACEA of patients in the study group after surgery was smaller than that of the control group (*P* < 0.05). It indicated that acromioplasty significantly increased the postoperative AT angle and decreased the ACEA, which might decrease the risk of postoperative rotator cuff reinjury. The above conclusions further confirmed the significance of acromioplasty. However, it is important to note that acromioplasty may lead to shoulder instability when there is a huge rotator cuff tear or a hard-to-repair rotator cuff injury [23]. Therefore, in order to further ensure the effectiveness of the combined surgical plan, care should be taken in performing acromioplasty, and the evaluation of shoulder function should be perfected before surgery. In addition, there was 1 postoperative infection in the study group. This suggests that we need to suture the injury according to the patient's condition and strengthen postoperative care to prevent the occurrence of postoperative infection.

In summary, arthroscopic acromion plasty and rotator cuff repair helped to promote the joint function recovery of aged patients with full-thickness rotator cuff tear combined with rotator cuff injury and alleviate the pain of the patients. Compared with simple rotator cuff repair, this technique can increase the postoperative AT and reduce the ACEA, and to some extent reduce the risk of postoperative rotator cuff reinjury, which is worthy of promotion. In addition, the shortcoming of this study lies in that, due to the trial time limit, a follow-up visit for a long time cannot be conducted in this study. In future relevant studies, the follow-up time should be appropriately extended in order to better observe and compare the clinical efficacy.

## Figures and Tables

**Table 1:** General information.

Group	Gender (*n*)		Age (years)	Course of disease (months)	Tearing length of rotator cuff (cm)	Affected side (*n*)	
	Male	Female				Left shoulder	Right shoulder
Study group (*n* = 42)	25	17	68.91 ± 3.45	6.73 ± 2.58	2.34 ± 0.75	19	23
Control group (*n* = 42)	24	18	68.78 ± 3.61	6.89 ± 2.41	2.31 ± 0.84	20	22
*t*/*χ*^2^	0.049		0.169	0.294	0.173	0.048	
*P*	0.825		0.866	0.770	0.863	0.827	

**Table 2:** Comparison of Constant–Murley and UCLA scores before and after surgery in two groups ($\bar{x}$ ± *S*, score).

Group	Constant–Murley		UCLA	
	Before surgery	After surgery	Before surgery	After surgery
Study group (*n* = 42)	73.20 ± 7.16	91.89 ± 3.64^a^	23.47 ± 3.69	32.05 ± 1.75^a^
Control group (*n* = 42)	73.52 ± 7.23	86.51 ± 6.33^a^	23.85 ± 3.73	29.96 ± 1.82^a^
*t*	0.204	4.775	0.469	5.365
*P*	0.839	<0.001	0.640	<0.001

Note: “a” is *P* < 0.05, compared with the same group before operation.

**Table 3:** Comparison of VAS scores of patients between the two groups before and at each time point after surgery ($\bar{x}$ ± *S*, score).

Group	Before surgery	2 weeks after operation	2 months after operation	6 months after operation
Study group (*n* = 42)	6.22 ± 1.41	4.23 ± 1.26^a^	3.10 ± 1.16^ab^	1.89 ± 0.98^abc^
Control group (*n* = 42)	6.29 ± 1.53	4.97 ± 1.33^a^	3.65 ± 1.27^ab^	2.25 ± 0.63^abc^
*t*	0.218	2.618	2.072	2.003
*P*	0.828	0.011	0.041	0.049

Note: “a” is *P* < 0.05, compared with that in the same group before surgery; “b” is *P* < 0.05, compared with that in the same group two weeks after surgery; “c” is *P* < 0.05, compared with that in the same group six months after surgery.

**Table 4:** Comparison of active range of motion between the two groups before and after surgery ($\bar{x}$ ± *S*,°).

Group	Anterior shoulder flexion		Abduction		Neutral external rotation		Abduction 90 internal rotation		Abduction 90 external rotation	
	Before surgery	After surgery	Before surgery	After surgery	Before surgery	After surgery	Before surgery	After surgery	Before surgery	After surgery
Study group (*n* = 42)	80.13 ± 11.86	160.45 ± 5.37^a^	76.25 ± 5.66	162.53 ± 7.11^a^	24.96 ± 5.28	43.33 ± 3.19^a^	63.22 ± 6.28	84.14 ± 4.11^a^	66.19 ± 4.73	84.15 ± 3.41^a^
Control group (*n* = 42)	81.14 ± 11.52	155.74 ± 5.63^a^	76.79 ± 5.81	157.58 ± 6.34^a^	24.75 ± 5.31	40.39 ± 3.41^a^	63.58 ± 6.31	80.19 ± 3.52^a^	67.14 ± 4.52	80.17 ± 3.59^a^
*t*	0.396	3.923	0.432	3.368	0.182	4.080	0.262	4.731	0.941	5.209
*P*	0.693	<0.001	0.667	0.001	0.856	<0.001	0.794	<0.001	0.349	<0.001

Note: “a” is *P* < 0.05, compared with the same group before operation.

**Table 5:** Comparison of morphological parameters of acromion between the two groups before and after surgery ($\bar{x}$ ± *S*, °).

Group	CSA		At		LAA		AI		ACEA	
	Before surgery	After surgery	Before surgery	After surgery	Before surgery	After surgery	Before surgery	After surgery	Before surgery	After surgery
Study group (*n* = 42)	42.52 ± 3.63	32.17 ± 2.29^a^	32.24 ± 5.47	35.29 ± 4.19^a^	67.59 ± 7.84	66.72 ± 5.34^a^	0.69 ± 0.09	0.69 ± 0.02^a^	18.79 ± 2.41	15.53 ± 2.28^a^
Control group (*n* = 42)	42.37 ± 4.17	33.49 ± 2.18^a^	32.15 ± 5.67	34.38 ± 4.27^a^	67.83 ± 7.53	66.90 ± 5.41^a^	0.69 ± 0.08	0.69 ± 0.01^a^	18.63 ± 2.57	16.94 ± 2.71^a^
*t*	0.176	2.706	0.074	0.986	0.143	0.154	0.000	0.000	0.294	2.580
*P*	0.861	0.008	0.941	0.327	0.887	0.878	0.001	1.000	0.769	0.012

Note: “a” is *P* < 0.05, compared with the same group before operation.

**Table 6:** Comparison of surgical indexes between the two groups ($\bar{x}$ ± *S*).

Group	Operation time (min)	Blood loss (mL)	Incision length (cm)	Length of hospital stay (d)
Study group (*n* = 42)	92.15 ± 10.52	23.79 ± 4.75	4.53 ± 0.31	5.47 ± 1.12
Control group (*n* = 42)	89.43 ± 11.16	22.98 ± 4.66	4.47 ± 0.32	6.69 ± 1.25
*t*	1.149	0.789	0.873	4.712
*P*	0.254	0.433	0.385	<0.001

## Data Availability

The data used and/or analyzed during the current study are available from the corresponding author.
